# The Combined Clinical Efficacy and Safety Analysis of Adoptive Immunotherapy with Radiotherapy and Chemotherapy in Non-Small-Cell Lung Cancer: Systematic Review and Meta-Analysis

This article has been retracted.

**DOI:** 10.1155/2022/2731744

**Published:** 2022-06-06

**Authors:** Zhiming Fan, Honggui He, Liqun Chen

**Affiliations:** Departments of Oncology, The First Naval Hospital of Southern Theater of People's Liberation Army, Zhanjiang, Guangdong, China

## Abstract

**Objective:**

To explore the differential efficacy of chemoradiotherapy combined with adoptive immunotherapy and radiochemotherapy alone in patients with non-small-cell lung cancer (NSCLC).

**Methods:**

Qualified randomized controlled trial (randomized controlled trial, RCT), or nonrandomized concurrent controlled trial (NRCCT), published in various databases, including PubMed, EMBASE, Chinese journal full-text database, Medline, Cochrane database, and VIP Chinese database, and the Revman5. 0 software performed the data analysis.

**Results:**

We found the significantly different curative effect between the experimental and control groups (OR = 1.94, 95% CI (1.46, 2.58), *P* < 0.001, *I*^2^ = 0%, *Z* = 4.59), effect of adoptive immunotherapy on the progression of disease (OR = 1.80, 95% CI (1.38, 2.35), *P* < 0.001, *I*^2^ = 0%, *Z* = 4.33), adoptive immunotherapy on overall survival (OR = 2.19, 95% CI (1.60, 2.99), *P* < 0.001, *I*^2^ = 0%, *Z* = 4.91), and adverse effects of adoptive immunotherapy (OR = 1.76, 95% CI (1.25, 2.48), *P* = 0.001, *I*^2^ = 0%, *Z* = 3.26).

**Conclusion:**

Adoptive immunotherapy combined with microradiotherapy can decrease the recurrence of NSCLC and improve patient survival, as well as early patients can be benefited more significantly from immunotherapy.

## 1. Introduction

In the world, lung cancer is a leading malignant tumor with a significant number of diagnosed and dead people. Every year, about 1.6 million diagnosed people and 1.37 million people die from lung cancer, while 85% of lung cancer cases included non-small-cell lung cancer (NSCLC) cases [1–3]. In resectable and unresectable lung cancer patients, systemic therapy combined with local therapy has improved the prognosis better [4]. But even in combination with postoperative adjuvant chemoradiotherapy, more than 40% of patients will be relapsed which in turn leads to death [5], while tumor immunotherapy can be associated with removing the residual lesions, inhibiting the recurrence in the postoperative stage, correlated with a better survival rate of patients [6].

The malignant degree of cellular lung cancer is very high, not only the deterioration rate is very fast, but also the invasion intensity is very large, and the clinical treatment is usually routine with highly sensitive radiotherapy and chemotherapy [7]. However, it should not be ignored that chemoradiotherapy is prone to drug resistance, which will greatly reduce the therapeutic effect of chemoradiotherapy on small-cell lung cancer, and is not suitable to treat the non-small-cell lung cancer. In recent decades, tumor immunotherapy has flourished, and various treatment options have emerged. Adoptive immunotherapy refers to the in vitro expansion of various tumor-killing cells, including lymphokine-activated killer cell (LAK) which is activated by various lymphokines, tumor-infiltrating lymphocyte (TIL), and cytokine-induced killer cells (CIK). There are an increasing number of clinical trials for treating solid tumors, including liver cancer and lung cancer [8].

To improve the clinical curative effect, efficient and safe cellular immunotherapy is often used as adjuvant therapy [9]. In the course of radiotherapy and chemotherapy, patients will have some complications, nausea, vomiting, and other organ function damage, which will affect the recovery of the patient's disease. To reduce the treatment confidence of patients, it is crucial to choose an effective treatment method which can reduce the rate of complications. With the development and progress of medical technology in China, the use of biological immunotherapy combined with chemoradiotherapy to treat this type of patient has appeared clinically [10].

In this study, we identified whether adoptive immunotherapy or chemoradiotherapy can reduce the recurrence rate of lung cancer patients and improve the survival rate. Also, we evaluate the safety of their application for treating non-small-cell lung cancer.

## 2. Materials and Methods

### 2.1. Data Source

We searched PubMed, EMBASE, Chinese journal full-text database, Medline, Cochrane database, and VIP Chinese database from January 1995 to September 2021. For all the retrieved pieces of literature, references were searched and read, and methods such as literature tracing and manual literature searching were adopted to ensure the completeness of the pieces of literature. The restricted languages were English and Chinese literatures. We used numerous subject words in the literature retrieval process, including “lung cancer”, “non-small cell lung cancer”, “small cell lung cancer”, “immunotherapy in lung cancer”, “chemo-radiotherapy”, “cytotoxic T lymphocyte”, “lymphokine-activated killer cell”, “tumor Infiltrating lymphocyte”, “cytokine-induced killer cell”, “Gamma-delta T cell”, “clinical trial of lung cancer”, “Adoptive cell therapy in cancer”, “RCT”, “adoptive immunotherapy”, “non-trivial cellular lung cancer”, “CIK”, “LAK”, and “TILs”. We used Noteexpress software to manage related literature and eliminated the duplication of literature (Figure 1).

### 2.2. Inclusion Criteria for Literature Data

(1) Research type: literature published at home and abroad from January 1995 to September 2021, covering randomized controlled trial (RCTS) or nonrandomized concurrent controlled trials (NRCCT) of adoptive immunotherapy in NSCLC, and the mean follow-up time was at least 2 years; (2) subjects: patients diagnosed with NSCLC by pathology or multiple imaging examinations, regardless of age, race, nationality, or gender; (3) intervention measures: radiotherapy and chemotherapy combined with adoptive immunotherapy in the treatment group and radiotherapy and chemotherapy alone in the control group; and (4) study endpoint events, patient death, tumor recurrence, or metastasis.

### 2.3. Exclusion Criteria for Literature Data

(1) Abstract, case reports, comments, and review; (2) repeated reports, poor report quality, little reporting information, unclear data description, and special sample selection; (3) no research comparing two treatment plans; (4) repeated research by the same research unit, excluding old documents; and (5) documents with small sample size (*n* < 20).

### 2.4. Estimation of Quality

To judge whether there is bias and its influence degree, the quality of the included literature is evaluated from the following aspects: (1) whether the inclusion criteria and basic composition characteristics of the research objects are accurate; (2) whether the experimental design is reasonable; (3) whether the statistical method is appropriate; and (4) whether the bias in this study is discussed. The evaluation process is completed independently by the two reviewers, and the inconsistency will be solved through discussion. If there is still a dispute, please make an expert comment.

### 2.5. Data Extraction

The two researchers extracted the literature-related data, respectively, and the data extraction table included the authors, reporting time, pathological stage, treatment plan, drugs, grouping method and number of people, survival rate, and time without progression.

### 2.6. Statistical Analysis

We employed RevMan5.0 software for computational analysis. Studies with good homogeneity by heterogeneity test (*P* > 0.1) were analyzed by the fixed-effect model, whereas we analyze the data by the random effect model. The statistical data were calculated with an odds ratio (OR) and 95% CI. When *P* < 0.05 and 95% CI did not include 1, the difference in point estimates of OR was considered statistically significant. Weighted mean difference and 95% CI were calculated for measurement data. A funnel plot was drawn to analyze publication bias.

## 3. Result

### 3.1. Retrieved Results

According to the search keywords, 99 related works of literature were found, including 73 English literature, 26 Chinese literature, and 30 duplicate literature. Referring to the inclusion and exclusion criteria of kinds of literature, 25 pieces of literature with unavailable or incomplete data and 34 literatures with poor research quality and unqualified data were excluded after searching one by one. A total of 12 works of literatures [11–22] were screened for meta-analysis, and there were no significant differences in age, gender, stage, and other aspects of patients in the included pieces of literature (*P* > 0.05). The characteristics and situations of each study are shown in Table 1.

### 3.2. Curative Effect

We included the 12 RCT kinds of literature in curative effect. We applied the heterogeneity test, and we found that the selected studies have small heterogeneity. Therefore, we performed the meta-analysis with fixed models. In the meta-analysis, the rhombus plot and vertical line did not intersect in the forest map of curative effect for the 4 included studies, which indicated the significant difference in curative effect between the experimental and control groups (OR = 1.94, 95% CI (1.46, 2.58), *P* < 0.001, *I*^2^ = 0%, *Z* = 4.59) (Figure 2).

### 3.3. Effect of Adoptive Immunotherapy on Disease Progression

We included the 12 RCT pieces of literatures to evaluate the effect of adoptive immunotherapy on disease progression. We applied the heterogeneity test, and we found that the selected studies have small heterogeneity. Therefore, we performed the meta-analysis with fixed models. In the meta-analysis, the rhombus plot and vertical line did not intersect in the forest map of effect of adoptive immunotherapy on disease progression for the included 4 previous studies, which indicated the significant difference in the effect of adoptive immunotherapy on disease progression between the experimental and control groups (OR = 1.80, 95% CI (1.38, 2.35), *P* < 0.001, *I*^2^ = 0%, *Z* = 4.33) (Figure 3).

### 3.4. Effects of Adoptive Immunotherapy on Overall Survival

We included the 12 RCT pieces of literature to evaluate the effect adoptive immunotherapy on overall survival. We applied the heterogeneity test, and we found that the selected studies have small heterogeneity. Therefore, we performed the meta-analysis with fixed models. In the meta-analysis, the rhombus plot and vertical line did not intersect in the forest map of effect of adoptive immunotherapy on overall survival for the included 4 pieces of literature, indicating the significant difference of the effect of the adoptive immunotherapy on overall survival between the experimental and control groups (OR = 2.19, 95% CI (1.60, 2.99), *P* < 0.001, *I*^2^ = 0%, *Z* = 4.91) (Figure 4).

### 3.5. Adverse Effects of Adoptive Immunotherapy

We included the 12 RCT pieces of literature to evaluate the adverse effects of adoptive immunotherapy. We applied the heterogeneity test, and we found that the selected studies have small heterogeneity. Therefore, we performed the meta-analysis with fixed models. In the meta-analysis, the rhombus plot and vertical line did not intersect in the forest map of effect of adverse effects of adoptive immunotherapy for the included 4 studies, indicating the significant difference in adverse effects of adoptive immunotherapy between the experimental and control groups (OR = 1.76, 95% CI (1.25, 2.48), *P* = 0.001, *I*^2^ = 0%, *Z* = 3.26) (Figure 5).

### 3.6. Published Bias Analysis

Use RevMan5. 0. The inverted funnel plot was drawn by a software, and the funnel plot was symmetric, indicating that the heterogeneity in this study was not significant (Figures 6 and 7).

## 4. Discussion

In the tumor microenvironment, adoptive immunotherapy included various immune cells which are associated with antitumor effects. Some of these cells included the LAK, TILs, cytotoxic T cells (CTL)), CIK, and T cells [23–25]. LAK cells are a class of killer cells induced by peripheral blood lymphocytes after IL-2 culture in vitro. TILs are lymphocytes isolated from tumor tissue produced by IL-2 culture and CIK cells. Monocytes in peripheral blood are incubated by various cytokines, including CD3 monoclonal antibodies, IFN, or IL-2 [26]. CTL is a T cell loaded with a specific tumor antigen, and tumor cells are specifically identified and killed back in vitro [27–30]. T cells are a T cell that is not MHC limiting and is a class of immune cells recently used in various solid tumors. In recent years, adoptive immunotherapy is gradually accepted and recognized for treating various tumors [31]. To investigate the influence of tumor immunotherapy, the progression-free survival and overall survival of patients should be used as the most important indicator of the evaluation. Early patients have good immune status, and postoperative adoptive immune cells more thoroughly eliminate residual tumor cells and improve the survival time [32]. For advanced levels of patients, combined adoptive immunotherapy is crucially associated with the improvement of patients' immunological activities, especially after reducing postoperative tumor burden. Therefore, the early treatment of adoptive immunotherapy after reducing the tumor load can benefit the patients to a greater extent. In addition, patients who received CIK more than seven times were significantly better than those with fewer treatments [33].

Meta-analysis is a quantitative evaluation of controversial treatments. Meta-analysis is not only the best method to apply in RCTs but also an effective method for quantitative evaluation of existing outcomes in the absence of prospective randomized comparative trials [34]. Meta-analysis is an observational study, and bias is inevitable in the study design, collection of data, and computational analysis. Considering that the research articles with positive results may be more easily published than those with no positive results or negative results, which may lead to the bias of publication, in order to reduce publication bias, this study collected relevant literatures as comprehensively as possible through various ways and eliminated the repetitive short literatures [35]. The types of adoptive immune cells used and included in this study and the treatment regimens used in combination were different, so the results of the study were affected to some extent [36].

Immunotherapy methods for lung cancer are constantly innovating, and many clinical trials of immunological cytokines and vaccines for cancers are booming. A new meta-analysis revealed that the cytokines, vaccines for tumors, and monoclonal antibodies can positively affect patients with progressive NSCLC [37–39]. However, adoptive cell treatment does not have the uncertainty of whether effector cells have effective activation in vivo, and it is not accompanied by severe toxic reactions [40]. Altogether, adoptive immunotherapy gradually becomes a crucial measure for improving the survival rate of lung cancer patients. The researcher can hope for designing and developing numerous samples in the future. Multicenter RCT thus draws more reliable conclusions and guides the clinical treatment.

## Figures and Tables

**Figure 1:** Selecting and arranging the literature by using multiple databases and multiple subject words and arranging it into a flow chart.

**Figure 2:** Meta-analysis of efficacy comparison between experimental group and control group in non-small-cell lung cancer.

**Figure 3:** Meta-analysis of the effect of adoptive immunotherapy on disease progression in experimental group and control group in non-small-cell lung cancer.

**Figure 4:** Meta-analysis of the effect of adoptive immunotherapy on overall survival between two groups.

**Figure 5:** Meta-analysis of adverse reactions of adoptive immunotherapy in experimental group and control group in non-small-cell lung cancer.

**Figure 6:** The evaluation chart of literature quality. (a) Risk level of bias graph. (b) Risk level of bias summary.

**Figure 7:** (a) The funnel plot identifying the biased literature publication. (b) The funnel plot identifying the biased literature publication. (c) The funnel plot identifying the biased literature publication. (d) The Funnel plot identifying the biased literature publication.

**Table 1:** The basic clinical characteristics which are included in the selected 12 works of literature.

Name of studies	Age	Types of tumor	The experimental group (*N ***)**	Control group (*N ***)**	NOS score	Research type
Simone CB (2020)	63.71 ± 2.2	Lung tumor	75/120	52/120	8	RCT
Welsh J (2020)	55.65 ± 3.4	Lung tumor	68/102	41/101	7	RCT
Chen D (2020)	63.12 ± 4.5	Lung tumor	135/250	98/250	8	RCT
Theelen WSME (2021)	67.15 ± 4.5	Lung tumor	45/56	33/56	8	RCT
Peters S (2022)	52.85 ± 8.4	Lung tumor	61/88	55/88	8	RCT
Spigel DR (2022)	64.36 ± 10.2	Lung tumor	67/110	46/110	7	RCT
Verma V (2018)	62.62 ± 2.2	Lung tumor	46/78	35/78	9	RCT
Pakkala S (2020)	62.61 ± 3.0	Lung tumor	33/47	25/47	9	RCT
Ma SC (2021)	67.25 ± 4.5	Lung tumor	45/69	32/69	7	RCT
Twardowski P (2019)	66.22 ± 5.2	Lung tumor	80/112	66/112	8	RCT
Schoenfeld JD (2022)	61.35 ± 7.1	Lung tumor	105/150	90/150	9	RCT
Olkowski ZL (1978)	61.25 ± 6.1	Lung tumor	55/62	48/62	9	RCT

## Data Availability

The data used to support this study are available from the corresponding author upon request.
